# Hypoxia Regulates BMP4 Expression in the Murine Spleen during the Recovery from Acute Anemia

**DOI:** 10.1371/journal.pone.0011303

**Published:** 2010-06-24

**Authors:** Dai-Chen Wu, Robert F. Paulson

**Affiliations:** 1 Graduate Program in Biochemistry, Microbiology and Molecular Biology, The Pennsylvania State University, University Park, Pennsylvania, United States of America; 2 Department of Biochemistry and Molecular Biology, The Pennsylvania State University, University Park, Pennsylvania, United States of America; 3 Center for Molecular Immunology and Infectious Disease, The Pennsylvania State University, University Park, Pennsylvania, United States of America; 4 Department of Veterinary and Biomedical Sciences, The Pennsylvania State University, University Park, Pennsylvania, United States of America; Texas A&M University, United States of America

## Abstract

**Background:**

Bone marrow erythropoiesis is primarily homeostatic, producing new erythrocytes at a constant rate. However at times of acute anemia, new erythrocytes must be rapidly produced much faster than bone marrow steady state erythropoiesis. At these times stress erythropoiesis predominates. Stress erythropoiesis occurs in the fetal liver during embryogenesis and in the adult spleen and liver. In adult mice, stress erythropoiesis utilizes a specialized population of stress erythroid progenitors that are resident in the spleen. In response to acute anemia, these progenitors rapidly expand and differentiate in response to three signals, BMP4, SCF and hypoxia. In absence of acute anemic stress, two of these signals, BMP4 and hypoxia, are not present and the pathway is not active. The initiating event in the activation of this pathway is the up-regulation of BMP4 expression in the spleen.

**Methodology/Principal Findings:**

In this paper we analyze the regulation of BMP4 expression in the spleen by hypoxia. Using stromal cell lines, we establish a role for hypoxia transcription factor HIFs (Hypoxia Inducible Factors) in the transcription of BMP4. We identified putative Hypoxia Responsive Elements (HREs) in the BMP4 gene using bioinformatics. Analysis of these elements showed that in vivo, Hif2α binds two cis regulatory sites in the BMP4 gene, which regulate BMP4 expression during the recovery from acute anemia.

**Conclusions and Significance:**

These data show that hypoxia plays a key role in initiating the BMP4 dependent stress erythropoiesis pathway by regulating BMP4 expression.

## Introduction

Acute blood loss leads to tissue hypoxia, which induces a systemic response designed to increase oxygen availability to the tissues. Increased erythropoiesis is part of this response. Under steady state conditions, the bone marrow produces new erythrocytes at a constant rate to maintain homeostasis. In response to acute anemia stress, new erythrocytes must be rapidly produced. At these times stress erythropoiesis is the predominant form of erythropoiesis[1]. Stress erythropoiesis relies on a specialized population of stress erythroid progenitors that are primarily resident in the spleen[2]. These cells possess the ideal properties of stress response cells in that they are rapidly mobilized in response to acute anemia and are able to generate larger numbers of new erythrocytes much faster than bone marrow steady state erythroid progenitors[2], [3].

Three signals regulate the expansion of stress erythroid progenitors in the spleen, BMP4, SCF and hypoxia[3]. BMP4 acts on an immature cell, the BMP4 responsive cell (BMP4^R^), which causes it to differentiate into stress BFU-E. BMP4 also acts in concert with SCF and hypoxia to promote the proliferation and differentiation of stress BFU-E. Hypoxia plays a key role in this process by altering the response of progenitor cells to the other signals, which maximizes the expansion and differentiation of stress erythroid progenitors[3]. Acute anemia results in the complete mobilization of stress progenitors in the spleen. Following recovery, these progenitors are replenished by bone marrow cells that migrate into the spleen. Indian Hedgehog (Ihh) and Desert Hedgehog (Dhh) in the spleen induce the bone marrow progenitor cells to adopt the stress erythroid progenitor cell fate, which makes them competent to respond to BMP4 in response to acute anemia[4].

The BMP4 dependent stress erythropoiesis pathway has the potential to rapidly produce large numbers of new erythrocytes. Inappropriate activation of this pathway could result in polycythemia and lead to pathological consequences. However in the absence of anemic stress, this pathway is quiescent. Two levels of control maintain the pathway in the inactive state. Our previous work demonstrated that three signals are required for the expansion of stress progenitors, BMP4, SCF and hypoxia. Of these three signals only SCF is constitutively expressed in the spleen[3]. Tissue hypoxia is present only in response to anemia, and BMP4 expression is also limited to times of anemia. In our original analysis of this pathway, we proposed that BMP4 may be regulated by hypoxia[2]. This hypothesis would support the idea that anemic stress leading to tissue hypoxia would regulate two of the three signals needed for the expansion and differentiation of stress erythroid progenitors.

Hypoxia regulates gene expression primarily through the action of a family of transcription factors referred to as Hypoxia Inducible Factors or HIFs (for review see[5], [6], [7]). These transcription factors are made up of two subunits, an α subunit (Hif1α, Hif2α or Hif3α) which is stable under hypoxic conditions but rapidly degraded at normal O_2_ levels, and a β subunit (Hifβ or Arnt) that is unaffected by changes in O_2_ concentration. The HIF complex binds to a Hypoxia Responsive Element (HRE), where it recruits co-activators p300/CBP to promote gene transcription[8]. At normal levels of O_2_, the α subunits are hydroxylated on a proline residue by a family of proline hydroxylases (PHDs)[9], [10], [11], [12]. The hydroxylated proline is recognized by the product of the von Hippel Lindau tumor suppressor gene, VHL, which targets the protein for ubiquitination and destruction. At low levels of O_2_, the PHDs are inhibited and the α subunits are stable. The interaction of HIF with co-activators is also regulated by O_2_ concentration. FIH-1 is an asparaginyl hydroxylase which functions at moderate to high O_2_ levels[13], [14], [15]. Asparagine hydroxylated HIF is stable, but cannot bind co-activators, which allows for fine tuning of the hypoxia response. Hif1α[16], [17] and Hif2α[18], [19], [20] have been shown to be involved in the regulation of erythropoiesis. The analysis of targeted mutations of Hif1α or Hif2α or in genes that affect the stability of these molecules (*Vhl* [21] and *PHD2* [22]) showed that these mutations cause defects in murine erythropoiesis. The central role of this pathway in regulating erythropoiesis was further underscored by the identification of patients with erythrocytosis that have mutations in *PHD2* [23] and *HIF2*α[24], [25], [26] and the demonstration that Chuvash Polycythemia was caused by mutations in *VHL* [27], [28].

In this report, we have characterized the hypoxia dependent regulation of BMP4 expression during the recovery from acute anemia. We demonstrate that BMP4 expression is regulated at the transcriptional level by HIF. Using bioinformatics we identified five putative HREs and show that two of these potential regulatory sequences are bound by HIF *in vitro* and *in vivo*. Our data also show that *in vivo* during the recovery from acute anemia, Hif2α is the primary regulator of BMP4 expression in spleen.

## Materials and Methods

### Cell culture, mice and phenylhydrazine treatment

Murine spleen stromal cell line MSS31[29] (Japan Health Sciences Foundation, Health Science Research Resources Bank, Osaka Japan) was cultured in Gibco IMDM (Invitrogen, Carlsbad, CA) plus 10% fetal bovine serum (Equitech-Bio, Kerrville, TX), Penicillin-Streptomycin, 10 ug of transferrin, 0.2 g of BSA, 1 mg of insulin, and 10 ug of EGF. Murine bone marrow stromal cell line W2017[30] (American Type Culture Collection, Manassas, VA) was cultured in Gibco DMEM (Invitrogen, Carlsbad, CA) plus 10% fetal bovine serum (Equitech-Bio, Kerrville, TX), Penicillin-Streptomycin, and 1.5 g of Na_2_CO_3_. Murine fetal liver stromal cell line AFT024[31] (American Type Culture Collection, Manassas, VA) was cultured in Gibco DMEM (Invitrogen, Carlsbad, CA) plus 10% fetal bovine serum (Equitech-Bio, Kerrville, TX), Penicillin-Streptomycin, 1.5 g of Na_2_CO_3_, and 0.05 mM beta-mercaptoethanol. HEK293T cells were cultured in Gibco DMEM (Invitrogen, Carlsbad, CA) plus 10% fetal bovine serum (Equitech-Bio, Kerrville, TX), and Penicillin-Streptomycin. C57BL/6 mice (Jackson Laboratory, Bar Harbor, ME) were approximately 6 to 8 weeks old, and controls were matched for gender and age. Acute anemia was induced by injection of phenylhydrazine (Sigma, St Louis, MO) at the concentration of 100 mg/kg mouse in phosphate-buffered saline (PBS) buffer. All procedures using mice were approved by the IACUC of the Pennsylvania State University (IACUC Protocol #30584).

### Transfection of shRNA

shRNA plasmids target for Hif1α, Hif2α, GATA2 (served as control) (TCR3-54449, TCR3-54450, TCR3-82303, TCR3-82306, TRC5-85419, Open Biosystem, Huntsville, AL) were transfected into HEK293T cells with TransIT®-293 transfection reagent (Mirus, Madison, WI).

### Prediction of potential HREs (HIF Responsive Elements)

Mouse BMP4 DNA sequence with 5000 extra bp upstream and 5000 extra bp downstream was gained from UCSC Genome Browser created by the Genome Bioinformatics Group of UC Santa Cruz, and analyzed with transcription factor analysis program MatInspector[32]. The acquired sequences data were as of Sep, 2005. The sequences of the predicted HREs were then aligned and the conservation among mammal species was compared for further selection of candidates.

### RT-PCR

Total RNA isolated from cell lines or spleen cells was homogenized in TriZol (Invitrogen, Carlsbad, CA) and reverse transcribed into cDNA by using SuperScriptII system (Invitrogen, Carlsbad, CA). BMP4 gene expression was determined with primers 5′-CCTGGTAACCGAATGCTGAT-3′ and 5′-TGTGATGAGGTGTCCAGGAA-3′;

β-actin gene expression was determined with primers 5′-AGCCATGTACGTAGCCATCC-3′ and 5′-TTTGATGTCACGCACGATTT-3′;

28s rRNA gene expression was determined with primers 5′-TTGAAAATCCGGGGGAGAG-3′and 5′-ACATTGTTCCAACATGCCAG-3′. Relative quantification of BMP4 expression was also determined by TaqMan probe using 18 s rRNA as the internal control (Applied Biosystems, Foster City, CA).

### Chromatin immunoprecipitation (ChIP) assay

Spleens were diced into small pieces and resuspended in phosphate-buffered saline (PBS) containing freshly added Complete Protease Inhibitor Cocktail (Roche, Indianapolis, USA) and homogenized. Cross-linking of proteins to the DNA of cells (isolated from spleen or cell culture) was achieved by adding formaldehyde to a final concentration of 1% for 15 min at 37°C with occasional inversion. Glycine was then added to a final concentration of 0.25 M, and the reaction was incubated at room temperature for 10 min with occasional inversion. Cells then were washed twice with ice-cold PBS containing freshly added protease inhibitors. Cell pellets were collected at 1000 rpm at 4°C. Cells were resuspended in SDS cell lysis buffer (50 mM Tris-HCl (pH 8.1), 10 mM EDTA, 1% SDS, and protease inhibitor) for 20 min on ice. For spleen cells, prior to further lysis by SDS cell lysis buffer, pellets were first resuspended in cell lysis buffer (5 mM PIPES [PH 8.0], 85 mM KCl, 0.5% NP-40, and protease inhibitor) for 20 min on ice. Cells were sonicated to give a DNA size range from 200 to 900 bp. Samples were centrifuged for 10 min at 13,000 rpm at 4°C to remove debris and the supernatants were transferred to new microcentrifuge tube. DNA concentration of each sample was measured to ensure an equal amount of DNA for further immunoprecipitation. 10 ug of samples were pre-cleared with salmon sperm DNA/protein A or G agarose slurry (Upstate Biotechnology, Lake Placid, NY) for 1 hr at 4°C with agitation and then spun down at 4°C at 2000 rpm. The supernatant fractions were collected and diluted 10-fold with dilution buffer (16.7 mM Tris-HCl, pH 8.1, 1.1% Triton X-100, 1.2 mM EDTA, 167 mM NaCl, 0.01% SDS, and protease inhibitor). 5 or 10% of each sample was kept as input control for PCR. Samples were incubated with antibodies overnight at 4°C. Immune complexes were collected using salmon sperm DNA/protein A or G agarose slurry for 1 hr at 4°C, and collected at 2000 rpm for 1 min. The samples were washed sequentially at 4°C with buffers as followings, low salt wash buffer (20 mM Tris-HCl (pH 8.1), 150 mM NaCl, 2 mM EDTA, 0.1% SDS, and 1% Triton X-100), high salt wash buffer (20 mM Tris-HCl (pH 8.1), 500 mM NaCl, 2 mM EDTA, 0.1% SDS, and 1% Triton X-100), LiCl wash buffer (10 mM Tris-HCl (pH 8.1), 0.25 M LiCl, 1% Nonidet P-40, 1% deoxycholate, and 1 mM EDTA), and Tris-EDTA buffer. Immuno complexes were extracted from the agarose slurry with freshly prepared elution buffer (1% SDS and 0.1 M NaHCO_3_) by rotating 15 min at room temperature. Cross-linking of samples was reversed by adding NaCl at final concentration of 0.3 M to the eluates and incubating at 65°C for 4 hr to 16 hr. Afterwards the samples were digested with proteinase K, and the DNA was extracted with phenol-chloroform-isoamyl alcohol, purified by ethanol precipitation and stored at −80°C. The antibodies used for immunoprecipitation were anti- HIF1α (NB100–105, Novus Biologicals, Littleton, CO), anti-HIF2α (NB100–122, Novus Biologicals, Littleton, CO), anti-p300 (N-15, Santa Cruz Biotechnology, Santa Cruz, CA), anti-IgG (SC-2025, SC-2027, Santa Cruz Biotechnology, Santa Cruz, CA), anti- GATA2 (H116, Santa Cruz Biotechnology, Santa Cruz, CA), anti- SCL (E-14, Santa Cruz Biotechnology, Santa Cruz, CA), anti- Smad4 (C-20, Santa Cruz Biotechnology, Santa Cruz, CA).

PCR was performed within linear range and PCR products were separated on agarose gels, and quantified using ImageQuant. The following primers were used for amplification of precipitated DNA. HRE-1(forward): TGTCGGCGCTGTAAAGAGACG; HRE-1(reverse): TTGTCCCCGCCTGCTCTGAG; HRE-2(forward): TCCATCACAATGTGACACGG; HRE-2(reverse): ACTACGTTTGGCCCTTCTGC; HRE-3(forward): CATTCAACCACCTACACATACCAC; HRE-3(reverse): GTCAAAATATATGATCAATATGGTCAAAAC; HRE-4(forward): GCAATACCAGCACCCTACTTG; HRE-4(reverse): GTTCCTGTTGCTCTGGCTTG. PCR is also performed by using primers amplifying *Glut-1* promoter region as previously described, which served as positive and specificity controls for ChIP by HIF1α[33].

### Plasmid constructs and luciferase assay

Regions spanning *Bmp4* HRE's-2 and -4 were amplified by PCR with the following primers, digested with restriction enzymes and ligated into plasmid MCSgLuc[34], HRE2PCRinsert(F): GGAGTTCTCGAGGCAACCCAATTATG; HRE2PCRinsert(R): ATGCGGCCGCTGAGGTAACGATC; HRE4PCRinsert(F): ACGTCTCGAGAACTCAGGAAAGAAG; HRE4PCRinsert(R): ATGCGGCCGCGTGCTGGGTGAA. Plasmid clones containing HRE-2 or HRE-4 were further mutated by using QuikChange Site-Directed Mutagenesis Kit (Stratagene, La Jolla, CA) according to manufacturer's instruction with the following primers, HRE2mut(F): GACCCACCAGGGCCAGTTTTTCAGAATCAGCCGATCG; HRE2mut(R): CGATCGGCTGATTCTGAAAAACTGGCCCTGGTGGGTC; HRE4mutbp(F): GAAAGCTCACCATGAGGCCTATTTTGGCAAATAATCAGC; HRE4mutbp (R): GCTGATTATTTGCCAAAATAGGCCTCATGGTGAGCTTTC. These Lusiferase constructs were co-transfected with Renilla plasmid which serves as transfection efficiency control into HEK293T cells. After culture, luciferase activity was detected by Dual-Luciferase Reporter Assay System (Promega, Madison, WI) according to manufacturer's instruction.

### Statistical analysis

P values were calculated by student's t-Test with two-tailed distribution and two-sample equal variance.

## Results

### Hypoxia regulates the transcription of BMP4

Our analysis of the recovery from acute hemolytic anemia showed that BMP4 expression was induced in the spleen and our initial analysis suggested that BMP4 expression was regulated by hypoxia[2]. In addition to the spleen, BMP4 is also expressed in the fetal liver during development, and the BMP4 dependent stress erythropoiesis pathway drives the expansion of stress erythroid progenitors in the fetal liver[35]. We tested whether hypoxia could induce BMP4 expression in spleen stromal cells (MSS31[29]), fetal liver stromal cells (AFT024[31]) and a murine osteoblast cells line (W-20-17[30]). In figure 1A, the data show that in all three cells lines, culturing cells under hypoxic conditions (1% O_2_) leads to an induction of BMP4 mRNA (Figure 1A). The expression of BMP4 in AFT024 cells decreased at 24 hours of hypoxia, suggesting that other factors in these stromal cells may feed back to turn off BMP4 expression.

**Figure 1:** Hypoxia induces the transcription of BMP4. (A) RT-PCR analysis of BMP4, Hif1α, Hif1β, Hif2α or β-actin (control) expression in the MSS31 spleen stromal cell line (top); BMP4 and 28S rRNA (control) in the W2017 osteoblast cell line (middle) and BMP4 and 28S rRNA (control) in the AFT024 fetal liver stromal cell line (bottom) at 20% O_2_ or 1% O_2_. BMP4 expression relative to 18S rRNA in these cell lines was also examined by quantitative RT-PCR. (B) MSS31 cells were treated with Actinomycin D (ActD) (1 ug/ml) for 30 minutes prior to shifting the culture to 1% O_2_. At the indicated times cells were harvested, RNA was isolated and the expression of BMP4 was determined by RT-PCR.

Hypoxia induced transcription is mediated by the HIF transcription factor complex. However other mechanisms such as increased mRNA stability could also account for the increase in BMP4 expression. We hypothesized that this up-regulation of BMP4 expression was due to an increase in transcription caused by the HIF complex, which is known to activate transcription under low O_2_ conditions. To test the hypothesis, we first examined whether increased BMP4 expression by hypoxia is regulated at the transcriptional level. MSS31 cells were cultured in media alone or media plus the transcription inhibitor actinomycin D (ActD), and incubated at 20% O_2_ for 30 minutes. Cells were then cultured either at 20%O_2_ or shifted to 1% O_2_. The cells were harvested and BMP4 expression was examined by RT-PCR. ActD abolished the ability of hypoxia to induce BMP4 expression, indicating hypoxia regulates BMP4 expression by increasing the transcription of the BMP4 gene (Figure 1B).

### Hif1α and Hif2α are required for BMP4 induction under hypoxia

HIF is a heterodimer composed of α subunit encoded by Hifα genes and β subunit encoded by *Arnt* genes. The β subunit is not affected by oxygen change; however α subunits are unstable in the presence of oxygen. The N-terminal activation domain (NTAD) and C-terminal activation domain (CTAD) of Hifα subunit can activate transcription when bound to DNA in complex with β subunit (For review see[6], [7], [11]). Under very low O_2_, HIF activates transcription in concert with the co- activator p300/CBP[8]. To date, many HIF targets have been identified, which contain HIF Responsive Elements (HREs)[11]. Previous work showed that *Arnt−/−* embryonic stem cells were defective in the development of hematopoietic progenitors[36] and mutations in *HIF2α*, *PHD2* and *VHL* all cause defects in erythropoiesis[6], [19], [20], [21], [23], [24], [25], [26], [27], indicating that hypoxia or the HIF complex regulates hematopoiesis and in particular erythropoiesis. Here, we hypothesize that the HIF complex is required for regulating BMP4 transcription in the spleen during the recovery from acute anemia. To verify this hypothesis, we knocked down HIF1α or HIF2α expression by using short hairpin RNA (shRNA). In Figure 2A, the data show that clone HIF1α-50 and clone HIF2α-06 were able to efficiently knock down expression of HIF1α and HIF2α, respectively. HEK293T cells were transfected with these shRNA expression vectors. 24 or 48 hours post transfection, the cells were incubated at 20% O_2_ or shifted to 1% O_2_ for 16 hours. The expression of HIF1α or HIF2α and BMP4 were determined by RT-PCR with the expression of 28S rRNA used as control. Under hypoxic (1% O_2_) conditions, expression of HIF1α, HIF2α, and BMP4 were induced in HEK293T cells transfected with control construct (Figure 2B). When cells were transfected with shRNA constructs targeting either HIF1α or HIF2α, expression of HIF1α or HIF2α were no longer increased under 1% O_2_, showing that the knock-down by shRNA was efficient. The knockdown of HIF1α led to a loss of BMP4 expression in hypoxic cultures, while a decrease in HIF2α led to decreased expression of BMP4 compared to control when cells were grown in hypoxic cultures (Figure 2B). These results demonstrate that HIF1α and HIF2α are required for inducing BMP4 expression under hypoxia.

**Figure 2:** HIF1α and HIF2α are required for BMP4 induction under hypoxia. (A) RT-PCR analysis of the expression of HIF1α or HIF2α in HEK293T cells transfected with the indicated shRNA constructs. (B) RT-PCR analysis of BMP4 expression at 20% or 1% O_2_ in HEK293T cells where HIF1α (left) or HIF2α (right) were knocked down with shRNAs.

### The *Bmp4* locus contains 5 putative HIF responsive elements (HREs)

Our previous work identified a putative HRE in the 3′ UTR of the *Bmp4* gene[2] (HRE-3 in Figure 3A). This element was highly conserved in mouse, human and rat *BMP4* genes. In addition to this element which is highly similar to the HRE found in the 3′end of the Erythropoietin gene, we also analyzed the sequence of the *Bmp4* locus for other putative HREs. We used MATInspector[32] to analyze the *Bmp4* gene and 5000 bp on either side of the gene. Four additional potential binding sites for HIF-1 and/or bHLH/PAS protein family were identified by MATInspector (HRE's-1, 2, 4, 5 in Figure 3A). We next analyzed whether these five sites were conserved among species (Figure 3B). Sequence conservation among species is one measure that can be used to identify bona fide regulatory sites. Statistical models have been developed that provide additional information. We analyzed each of the sites for their regulatory potential (RP) scores (Figure 3B). RP scores are computed from genome-wide alignments of human and other organisms which take into account the conservation, composition and short-pattern structure information[37], [38]. Regulatory potential analysis was used to generate ESPERR 7 species RP scores[39]. This analysis in addition to sequence conservation showed that putative HRE's 1–4 were potential candidates for hypoxia regulatory elements, while HRE-5 lacked sequence conservation and was not further examined by experiments.

**Figure 3:** Identification of putative HREs in the murine BMP4 gene. (A) Schematic diagram of the location of the 5 putative HREs in BMP4 locus with extra 5000 bp both upstream and downstream, where the transcription start site is located at 6102 bp. The acquired sequence data were from September 2005. (B) The sequences of the 5 putative HREs are aligned among mammals. Sequences in grey box are conserved among 6 species. Below each alignment is the ESPERR 7 species RP score for each nucleotide.

### Hif1α, Hif2α and the transcriptional co-activator p300 are associated with *Bmp4* HRE's 2 and 4 in response to hypoxia *in vitro*

In order to examine whether the predicted HREs in the *Bmp4* locus are associated with the HIF complex in a hypoxia dependent manner, we performed chromatin immunoprecipitation (ChIP) assays with antibodies against HIF1α, HIF2α and the co-activator p300. MSS31 cells were cultured at either 20% O_2_ or 1% O_2_ for 16 hours, and then harvested for ChIP assay. IgG and other isotype control antibodies were used as specificity controls for immunoprecipitation. PCR primer pairs amplifying around 200 bp spanning these predicted HREs were used to assess the binding of Hif1α, Hif2α and p300. 5% or 10% of input DNA from both culture conditions were served as positive control for PCR and quantification control. In addition, a well-known Hif1α target, *Glut-1*, was served as positive and specificity control for ChIP assay by Hif1α (Figure 4C)[33].

**Figure 4:** HIF and co-activator p300 are associated with BMP4 under hypoxia in MSS31 cells. The binding of Hif1α, Hif2α, and p300 to these sites was investigated by ChIP assay in MSS31 cells cultured at 20% O_2_ or 1% O_2_ for 16 hours. IgG or other antibodies served as controls. PCR were performed with primers amplify HRE-2 (A) and HRE-4(B). Representative gel data are shown. The relative intensity of PCR products normalized to the input lanes is shown by combining data from three to five individual ChIP assays. (C) Positive and specificity controls of ChIP with Hif1α were examined at *Glut-1* locus.

Among our four candidates, we found that two HREs were associated with HIF and p300 in a hypoxia dependent manner. HRE-2, which is located within exon 3 of the *Bmp4* gene, exhibited hypoxia specific binding of Hif2α and p300 (Figure 4A). HRE-4, which is located approximately 4 kb 3′ of exon 3, exhibited binding of Hif1α, Hif2α and p300 under hypoxic conditions. The association with Hif2α was stronger than Hif1α at the HRE-4 site (Figure 4B). When we analyzed binding at the HRE-1 and HRE-3 sites, no PCR products were detectable until we increased the template amount to tenfold greater than that used with HRE-2 and 4. The amount of the PCR product generated at HRE-1 and 3 was similar regardless of whether the cells were cultured at 20% O_2_ or 1% O_2_ for all antibodies used for immunoprecipitation, suggesting that the interaction was not hypoxia inducible and represented background binding (data not shown). These data show that Hif1α, Hif2α and the coactivator p300 are associated with BMP4 under hypoxia *in vitro*; demonstrating a mechanism whereby BMP4 is regulated by HIF under hypoxia.

### Hif2α and the co-activator p300 are associated with HRE's 2 and 4 in the spleen following phenylhydrazine- induced acute hemolytic anemia

BMP4 expression is up-regulated in the spleen 24 hours after treatment with Phenylhydrazine to induce acute anemia[2]. We next tested whether these putative HREs are bound by Hif1α, Hif2α and p300 *in vivo* during the recovery from acute anemia. Tissue hypoxia is one of the physiological characteristics of acute anemia; we hypothesized that BMP4 is induced in spleen by HIF after phenylhydrazine- induced anemia. Spleen cells were harvested from control mice or mice treated with phenylhydrazine for RNA extraction and ChIP assay. In figure 5A, the data show that BMP4 expression was induced in the spleen at 24 hours post phenylhydrazine injection. At HRE-2 and HRE-4, we observed an increase in Hif2α and p300 binding following anemia induction (Figure 5B–C). Overall, the intensity of PCR bands, as quantified by ImageQuant software and normalized with input controls, showed that the association of Hif2α with HRE's 2 and 4 was stronger than Hif1α in phenylhydrazine-treated mice when compared to control mice (Figure 5B–C). There was no detectable binding to HRE-1 site. There was very weak binding of Hif2α and p300 to HRE-3 site (data not shown). These data demonstrate a mechanism whereby BMP4 is regulated in stress erythropoesis. The Hif2α complex and the co-activator p300 are associated primarily with HRE's 2 and 4 in the *Bmp4* gene in murine spleen at 24 hours post phenylhydrazine treatment. This time corresponds to the time when BMP4 is induced, which initiates the expansion of stress erythroid progenitors[2].

**Figure 5:** Binding of HIF and p300 to the BMP4 locus is induced by anemia. (A) RT-PCR analysis of BMP4 or β-actin (control) expression in primary spleen cells isolated from mice at 24 hours post induction of acute hemolytic anemia with phenylhydrazine (PHZ) and untreated mice. (B) Spleen cells were analyzed by ChIP assay using anti- HIF1α, HIF2α, p300 or IgG antibodies. PCR was performed with primers amplify HRE-2 (B) and HRE-4(C). Representative gel data are shown. The relative intensity of PCR products normalized to the input lanes is shown by combining data from three individual ChIP assays.

### HRE's 2 and 4 can confer hypoxia dependent expression to a luciferase expression plasmid

Our ChIP analysis identified two HREs that were bound by the HIF complex and p300 both in MSS31 cells *in vitro* and in the spleen at 24 hours after treatment with phenylhydrazine. These data suggest that these sites mediate hypoxia dependent expression of BMP4; we next tested whether these sites could confer hypoxia dependent expression on an exogenous luciferase gene. We cloned 100 bp fragments spanning either HRE-2 or HRE-4 or altered versions where these HREs were mutated (Figure 6A) upstream of luciferase gene expressed from a minimal murine β-globin promoter[34]. The HRE-2, HRE-2mut, HRE-4 or HRE-4mut plasmids were co-transfected with Renilla plasmid respectively into HEK293T cells. 24–48 hours after transfection with the plasmids, cells were cultured at 20% O_2_ or shifted to 1% O_2_ for overnight. Both HRE-2 luciferase and HRE-4 luciferase exhibit significant hypoxia dependent increases in expression when compared to luciferase alone at 20% O_2_ (Figure 6B). The hypoxia dependent induction was approximately 2.7 fold greater in HRE-2 luciferase and approximately 1.8 fold greater in HRE-4 luciferase when compared to the hypoxia dependent induction of the MCSgLuc vector. In both cases mutation of the HRE abolished the hypoxia dependent induction of luciferase activity (Figure 6B), showing that these HRE's are required for hypoxia dependent luciferase induction. These data demonstrate that HRE's 2 and 4 are capable of conferring hypoxia dependent transcription to exogenous genes and they regulate BMP4 expression during the recovery from acute anemia.

**Figure 6:** HRE-2 and HRE-4 can confer hypoxia inducible expression to a luciferase gene. (A) Sequence of wildtype and mutated versions of HRE-2 and HRE-4. (B) Luciferase activity in HEK293T cells transfected with the indicated plasmids at 20% or 1% O_2_. The firefly luciferase activity is normalized with renilla luciferase expression. Fold increase in luciferase activity was normalized with the increase observed in the control plasmid set to 1.0. p value was calculated to compare the luciferase activity under 20% versus 1% O_2_. Each bar represents the average of three to twelve individual transfections.

## Discussion

Our data show that the expression BMP4 in the spleen during the recovery from acute anemia relies primarily on the recruitment of Hif2α and p300 to specific sites in the *Bmp4* locus. We identified two HREs that exhibit hypoxia inducible binding of Hif2α and p300 both *in vitro* in MSS31 cells and *in vivo* in the spleen during recovery from acute anemia; these HREs are capable of conferring hypoxia inducible transcription when placed upstream of a luciferase reporter gene. These data show that BMP4 expression is regulated directly by hypoxia in spleen stromal cells.

*Hif2α* mutant mice exhibit embryonic lethality in inbred strains of mice, which complicated analysis of the role of Hif2α in adult hematopoiesis[18]. However, crossing the null mutation onto a mixed F1 background allowed mutant mice to survive. Analysis of these mice showed that *Hif2α−/−* mice developed pancytopenia. Further analysis of this phenotype showed that transplanted *Hif2α−/−* bone marrow could effectively generate new progenitor cells leading to normal hematopoiesis in recipient mice. In contrast, transplant of control bone marrow into *Hif2α−/−* recipients recapitulated the pancytopenia phenotype, which demonstrates that Hif2α functions in the hematopoietic microenvironment[20]. The primary target of Hif2α appears to be erythropoietin, as treatment of mutant mice with exogenous erythropoietin can rescue the defect in erythropoiesis[19]. Similar results were observed using *Hif2α* conditional alleles[18]. In these experiments, treatment with exogenous Epo also rescued the erythropoietic defects associated with deletion of *Hif2α* in adults. Our data suggests that BMP4 should be added to the list of genes regulated by Hif2α in the spleen microenvironment.

The BMP4 dependent stress erythropoiesis pathway is not limited to the spleen. Analysis of splenectomized mice showed that the adult liver can also support stress erythropoiesis[40]. BMP4 is normally expressed by hepatocytes in the liver. The expression pattern within each liver acinus forms a gradient of expression that fits a known oxygen gradient[41]. Highest expression of BMP4 is associated with regions that contain the lowest levels of oxygen. Our present study suggests a model where, in response to acute anemia, expansion of the hypoxia zone in the liver acini leading to an expansion of Hif2α dependent expression of BMP4[40].

Our data show that HRE-2 and HRE-4 can directly regulate hypoxia dependent induction of BMP4 expression. However, several observations suggested that the regulation of BMP4 during the recovery from acute anemia may be more complex. Studies examining hypoxia dependent transcription of BMP4 in hepatocellular carcinoma cells (HCC) showed that HIF1α dependent regulation of BMP4 expression is indirect in these cells[42]. Hypoxia induces the HIF1α dependent expression of ETS1, which in turn induces BMP4 expression. The authors showed that HIF1α was required for the BMP4 induction by transfecting a dominant negative form of HIF1α, which abolished BMP4 expression. However this effect could be overcome by over-expression of ETS1. This paper examined one putative HRE in the promoter of the human *BMP4* gene, which bound HIF1α weakly in gel mobility shift assay and did not correspond to any of HREs we characterized in this study. Our analysis showed that HRE-2 and HRE-4 can confer hypoxia inducible expression of luciferase gene. This induction was completely abolished when the HRE was mutated, which demonstrates that ETS1 does not regulate BMP4 expression through these sites.

In addition to HIF, the role of other transcription factors that may act independently or in concert with HIF to regulate BMP4 expression during recovery from acute anemia is also indicated by our previous work. Hedgehog signaling induces BMP4 expression by bone marrow progenitor cells when they enter the spleen microenvironment[4]. This induction is independent of hypoxia. Furthermore, we observed that BMP4 expression is delayed in the spleens of *flexed-tail (f)* mutant mice during the recovery from acute anemia[2] and in the fetal liver of mutant embryos[35]. *f/f* mice have a mutant Smad5, which acts as a dominant negative form with the ability to inhibit the function of Smads1, 5 and 8, which are activated by BMP4[2], [43]. This observation suggests that Smad 1, 5 and/or 8 may function with Hif2α to regulate transcription of BMP4 in the spleen during the recovery from acute anemia. Further analysis will be needed to address this question.
